This article has been retracted.

# Up-Regulation of Sonic Hedgehog Contributes to TGF-β1-Induced Epithelial to Mesenchymal Transition in NSCLC Cells

**DOI:** 10.1371/journal.pone.0016068

**Published:** 2011-01-13

**Authors:** Ma'in Y. Maitah, Shadan Ali, Aamir Ahmad, Shirish Gadgeel, Fazlul H. Sarkar

**Affiliations:** 1 Department of Pathology, Karmanos Cancer Institute, Wayne State University, Detroit, Michigan, United States of America; 2 Division of Hematology/Oncology, Department of Internal Medicine, Karmanos Cancer Institute, Wayne State University, Detroit, Michigan, United States of America; Florida International University, United States of America

## Abstract

**Background:**

Lung cancer, especially non-small cell lung cancer (NSCLC) is the major cause of cancer-related deaths in the United States. The aggressiveness of NSCLC has been shown to be associated with the acquisition of epithelial-to-mesenchymal transition (EMT). The acquisition of EMT phenotype induced by TGF-β1in several cancer cells has been implicated in tumor aggressiveness and resistance to conventional therapeutics; however, the molecular mechanism of EMT and tumor aggressiveness in NSCLC remains unknown.

**Methodology/Principal Findings:**

In this study we found for the first time that the induction of EMT by chronic exposure of A549 NSCLC cells to TGF-β1 (A549-M cells) led to the up-regulation of sonic hedgehog (Shh) both at the mRNA and protein levels causing activation of hedgehog signaling. These results were also reproduced in another NSCLC cell line (H2030). Induction of EMT was found to be consistent with aggressive characteristics such as increased clonogenic growth, cell motility and invasion. The aggressiveness of these cells was attenuated by the treatment of A549-M cells with pharmacological inhibitors of Hh signaling in addition to Shh knock-down by siRNA. The inhibition of Hh signaling by pharmacological inhibitors led to the reversal of EMT phenotype as confirmed by the reduction of mesenchymal markers such as ZEB1 and Fibronectin, and induction of epithelial marker E-cadherin. In addition, knock-down of Shh by siRNA significantly attenuated EMT induction by TGF-β1.

**Conclusions/Significance:**

Our results show for the first time the transcriptional up-regulation of Shh by TGF-β1, which is mechanistically associated with TGF-β1 induced EMT phenotype and aggressive behavior of NSCLC cells. Thus the inhibitors of Shh signaling could be useful for the reversal of EMT phenotype, which would inhibit the metastatic potential of NSCLC cells and also make these tumors more sensitive to conventional therapeutics.

## Introduction

An estimated 1.35 million individuals were diagnosed with lung cancer worldwide in 2009. Lung cancer is the most common cause of cancer related mortality in the United States, with more than 160,000 deaths per year and 85% of all lung cancers are non-small cell lung cancer (NSCLC) [1]. Greater than 70% of NSCLC patients, at present, shows metastases to the regional lymph nodes or to distant sites [2]. While, systemic therapy plays a major role in the management of most NSCLC patients, the benefits of systemic therapy are modest. The median survival of NSCLC patients with distant metastases ranges from 9-12 months, with median progression free survival (PFS) of only 3.5 to 5.5 months. Therefore, there is an urgent need to develop novel therapies based on newer understanding of the molecular mechanisms and pathways that participate in lung carcinogenesis for better and improved treatment of patients diagnosed with NSCLC.

Emerging evidence suggests that the acquisition of epithelial-to-mesenchymal transition (EMT) phenotype could be induced by Transforming Growth Factor-β (TGF-β) especially TGF-β1 among other factors, resulting in tumor invasiveness, and these EMT-type cells have been classified as cancer stem-like cells in recent studies [3]. The importance of EMT process have been established in embryonic development [4]. Lately, EMT has also been found to play a critical role in tumor invasion, metastatic dissemination and the acquisition of resistance to conventional therapies [5]–[12]. Moreover, EMT phenotype in cancers has been associated with poor clinical outcome in multiple cancer types including NSCLC, yet the molecular mechanisms underlying the induction of EMT by TGF-β1 remain ill-defined especially for NSCLC [13]–[17].

Since the acquisition of an EMT phenotype has emerged as an important mediator of cancer progression, cancer metastases and resistance to both chemotherapy and targeted drugs such as EGFR inhibitors, thus further mechanistic studies to ascertain the role of TGF-β1- induced EMT are warranted. The clinical relevance of EMT and drug insensitivity comes from recent studies showing an association between epithelial markers and sensitivity to erlotinib in NSCLC cell lines [17]–[19], suggesting that EMT-type cells are resistant to erlotinib, however the role of signaling molecules in mediating the induction of EMT by TGF-β1 is lacking. Among the various molecular pathways, the Hedgehog (Hh) signaling pathway has emerged as an important mediator of carcinogenesis and cancer metastases [20], [21]. Studies have shown that the Hh signaling pathway, a pathway normally active in human embryogenesis and tissue repair, is also active in many cancers including NSCLC [22]–[25]. Hh inhibitors are now being tested in preclinical and clinical settings based on findings that the inhibition of Hh signaling could inhibit cell growth, invasion and metastasis of cancer cells [26]–[28]. The Hh signaling pathway is comprised of the ligand sonic, indian, and desert hedghog (Shh, Ihh, Dhh, respectivly), and the cell surface molecules Patched (PTCH) and Smoothened (SMO). In the absence of an Hh ligand, PTCH causes suppression of SMO [29], [30]; however, upon ligand binding to PTCH, SMO protein translocates into the primary cilium, and leads to the activation of transcription factor GLI1, which then translocates to the nucleus, leading to the expression of Hh target genes [29], [30]. GLI1-mediated expression of genes is involved in cell growth and differentiation [29], and thus the activation of Hh signaling is believed to play an important role in tumor cell invasion and metastasis.

Based on the above findings and the lack of mechanistic studies in establishing the role of TGF-β1-induced activation of Hh signaling with respect to the acquisition of EMT and tumor cell aggressiveness, we used NSCLC cells as a preclinical model for the current study. Here we show for the first time that chronic exposure of A549 cells (NSCLC cells) to TGF-β1 led to the acquisition of EMT phenotype with concomitant up-regulation of sonic hedgehog (Shh) both at the mRNA and at the protein levels, which is consistent with findings in another NSCLC cell line (H2030). The up-regulation of sonic hedgehog was consistent with increased cell motility, invasion, and tumor cell aggressiveness. In addition, we found that this process could be attenuated by Shh siRNA as well as by chemical inhibitors of Hh signaling such as cyclopamine and GDC-0449. Moreover, we found that the inhibition of Hh signaling by pharmacological inhibitors led to the reversal of EMT phenotype as confirmed by the reduction of mesenchymal markers such as ZEB1 and Fibronectin, and induction of epithelial marker E-cadherin, suggesting that the acquisition of EMT phenotype by TGF-β1 in NSCLC cells is mechanistically mediated by the activation of Shh signaling because the knock-down of Shh by Shh specific siRNA attenuated TGF-β1-induced EMT phenotype.

## Results

### Induction of epithelial-to-mesenchymal transition (EMT) in A549 NSCLC cells by chronic exposure to TGF-β1

It has been reported that A549 cells undergoes EMT phenotypic changes upon exposure to TGF-β1 [13], [14]. This was seen as trans-differentiation, especially because the exposure was done for a short period of time (48–72 hours). In an attempt to recapitulate the *in vivo* situation where cells are chronically exposed to TGF-β1 in the tumor microenvironment, we exposed A549 cells to TGF-β1 up to three weeks. After 21 days of exposure to TGF-β1, A549 cells morphology was found to be completely changed to a mesenchymal phenotype (we termed this cells as A549-M cells), with an elongated and disseminated appearance (Fig. 1A). To confirm the mesenchymal phenotype, we assessed the expression of molecular markers of EMT such as ZEB1 mRNA, which has been reported earlier to serve as a mesenchymal marker [31], [32], and we found that ZEB1 was up-regulated, while the expression of E-cadherin mRNA, an epithelial marker, was down-regulated (Fig. 1B). Fibronectin protein, a mesenchymal marker [17], was also found to be highly up-regulated in A549-M cells (Fig. 1C).

**Figure 1:** Induction of epithelial to mesenchymal transition (EMT) in A549 cells by chronic exposure to TGF-β1: TGF-β1 was added to A549 cells in culture media and maintained for 21 days with changing medium every third day with freshly added TGF-β1. A) Phase contrast objective microscopic pictures at 10× magnification. A549 cells morphology changed to mesenchymal phenotype (A549-M cells). Cell shape appears elongated and non-polarized. B) qRT-PCR of A549 and A549-M cells. A549-M cells showed a lower E-cadherin “epithelial marker,” and a higher ZEB1 “EMT marker”, at the mRNA levels. Delta-delta-CT was calculated, considering GAPDH as internal control and A549 parental as reference control. C) Western blot analysis where A549-M cells showed up-regulation of fibronectin “mesenchymal” marker compared to A549 parental cells.

### A549-M cells showed significant increase in cell migration and invasive characteristics compared to the A549 parental cells

Previous studies have shown that tumor cells with EMT phenotype are more motile [14], [17], [32], [33]. In order to further characterize A549-M cells, we performed a wound healing assay which showed increased cell migration of A549-M cells compared to parental cells (Fig. 2A). Moreover, we also found that A549-M cells are more invasive as documented by increased invasion as documented by matrigel-coated chamber assay (Fig. 2B), and A549-M cells also acquired more tumorigenic phenotype as documented by increased clonogenic growth (Fig. 2C).

**Figure 2:** A549-M cells shows significant increase in migration, invasive, and tumorigenic characteristics compared to A549 parental cells: TGF-β1-induced EMT phenotypic cells (A549-M cells) were generated as discussed under “Materials and Methods” section. A: showed wound healing assay results with its quantitative analysis. A549-M cells showed much higher motility compared to A549 parental cells. B and C showing the results of matrigel-coated membrane, and colony formation assays, respectively with its quantitative analysis. Significant increase was observed in the invasion and clonogenicity of A549-M cells compared to parental A549 cells. (*  =  *p*<0.05).

### A549-M cells showed up-regulation of sonic hedgehog mRNA, and protein expression

In order to assess the mechanism by which chronic TGF-β1 treatment induced EMT and tumor cell aggressiveness, we focused our investigation on Hh signaling because it has been implicated in EMT induction, metastasis and invasion [20]–[24], [26], [34], [34]–[37]. Interestingly, we found a dramatic increase in the expression of Hh pathway ligand Shh both at the mRNA and protein levels in A549-M cells whereas the parental A549 cells showed undetectable levels of Shh mRNA (Fig. 3A and Fig. 3B), which is consistent with published data showing that A549 parental cells contains undetectable levels of Shh expression [35]. In order to further confirm our findings documenting up-regulation of Shh by TGF-β1 treatment, and the induction of EMT in A549 NSCLC cell lines, we treated another NSCLC cell line (H2030 cells) with TGF-β1 for two weeks, and we found a significant increase in the expression of Shh mRNA, which was consistent with the induction of EMT marker ZEB1 and down-regulation of epithelial marker E-cadherin (Fig. 4A). These results suggest that TGF-β1 induced EMT is mediated by the transcriptional activation of Shh, which is the first such report in the literature.

**Figure 3:** A549-M cells showed up-regulation of sonic hedgehog (Shh) and GLI expression both at the mRNA and protein levels: A and B showing qRT-PCR and Western blot results, respectively for the expression of Shh whereas C and D represent the expression status of GLI at the mRNA and protein levels, respectively in A549-M cells compared to parental A549 cells. E represent Western blot data of GLI1 expression in NIH-3T3 cell after culturing with A549-M-derived conditioned media showing higher levels of GLI1 expression. (*  =  *p*<0.05).

**Figure 4:** Shh up-regulation is concomitant with TGF-β1-induced EMT in NSCLC cell lines. The up-regulation of Shh contributes to the EMT induction through TGF-β1. (A) H2030 cell line was treated with TGF-β1 (5 ng/ml) for two weeks, and the media was changed every three days. The qRT-PCR data showed induced expression of EMT marker ZEB1 mRNA, and reduced expression of epithelial marker E-cadherin mRNA, which was consistent with up-regulation of Shh mRNA similar to those observed in A549 cells exposed to TGF-β1. (B, C and D) A549 cells was transfected with Shh siRNA (A549-siShh) or scrambled siRNA (A549-si-ve) for 24 hrs prior to treatment with TGF-β1 (5 ng/ml) for 48 hrs, then the cells where collected for assays or re-transfected for the second time with siRNA or scrambled siRNA for 24 hrs (total 6days after siShh transfection) prior to the second time treatment with TGF-β1 (5 ng/ml) for another 48 hrs (total 5days of TGF-β1 treatment). (B) Upper panel shows transfection efficiency, and lower panel shows cellular morphology following treatments. A549-siShh maintained epithelial morphology after treatment with TGF-β1 at both time points as shown in left and right panels, respectively. (C) qRT-PCR expression of Shh mRNA showing significant down-regulation following Shh siRNA transfection (D) qRT-PCR expression of ZEB1 and E-cadherin mRNA. A549-si-ve cells showed down-regulation of epithelial marker, E-cadherin consistent with significant induction in the expression of ZEB1 as expected whereas TGF-β1 failed to show any effect on these markers in A549-siShh cells.

Interestingly, GLI1 levels in both A549-M and parental cells were higher compared to normal human bronchial epithelial cells (NHBE cells) although the expression of GLI1 was much more increased in A549-M cells (Fig. 3C and Fig. 3D). The high levels of Hh target gene GLI1 in both A549-M and A549 cells was observed despite the undetectable levels of Shh in A549 parental cells, which suggests that the expression of GLI1 could be ligand-independent in the parental A549 cells. Moreover, since Shh protein expression in A549-M cells appears to induce the GLI1 expression by an autocrine process, we further investigated this possibility using NIH-3T3 cells cultured with condition-media of A549-M cells. NIH-3T3 cells express Hh signaling receptor and transcription factor GLI1, and our data confirmed showing increased Hh signaling consistent with increased expression of GLI1 (Fig. 3E) in NIH-3T3 cells cultured with A549-M condition media. These results clearly show that A549-M cells secrete active Shh which can then activate Hh signaling in NIH 3T3 cells, resulting in the activation of GLI1. We further investigated the possibility whether Shh up-regulation directly mediates EMT induction by TGF-β1 or not. We found that knock-down of Shh by siRNA significantly attenuated TGF-β1 induced EMT, which was confirmed morphologically and molecularly as presented below. A549 cells transfected with Shh siRNA 24 hrs prior to treatment with TGF-β1 for 48 hrs (A549-siShh) maintained epithelial morphology, while scrambled siRNA (A549-si-ve) showed transformation to mesenchymal morphology (Fig. 4B left panel). Likewise, A549-si-ve showed more EMT induction compared to A549-siShh following re-transfection with Shh siRNA and treatment with TGF-β1 [Total six days of Shh siRNA transfection and five days after TGF-β1 treatment; details under figure legend (Fig. 4B right panel)]. The Shh siRNA trasfection resulted in significant knock-down of Shh expression as shown by qRT-PCR (Fig. 4C). We found significant attenuation in the induction of EMT by TGF-β1 treatment in A549 cells with Shh knock-down (A549-siShh cells) as confirmed by qRT-PCR. A549-si-ve cells showed down-regulation of epithelial marker, E-cadherin consistent with significant induction in the expression of ZEB1 as expected (Fig. 4D, 48 hrs TGF-β1) whereas TGF-β1 failed to show effect on these markers in A549-siShh cells. Moreover, we found further attenuation in EMT induction following second round of Shh siRNA transfection and TGF-β1 treatment. A549-si-ve cells showed a significant increase in ZEB1 expression consistent with significant down-regulation of E-cadherin (Fig. 4D, 5 days TGF-β1) whereas TGF-β1 failed to show effect on these markers in A549-siShh cells. These results demonstrated for the first time that Shh up-regulation by TGF-β1 is mechanistically linked with TGF-β1 induced EMT in NSCLC cells.

### Up-regulation of Shh in A549-M contributes to EMT-induced tumor cell migration and metastatic characteristics

Next, we investigated the role of increased expression of Shh in aggressive behavior such as migratory and metastatic potential of A549-M cells. We treated A549-M cells with Shh inhibitors such as cyclopamine and GDC-0449 and assessed their migration and invasion characteristics. Both cyclopamine and GDC-0449 significantly reduced cell migration and invasive capacity of A549-M cells (Fig. 5A–C and Fig. S1). Moreover, the treatment of A549-M cells by either cyclopamine (data not shown) or GDC-0449 showed partial reversal, where we observed incomplete attenuation of EMT phenotype, as documented by the reduced expression of fibronectin and ZEB1, and increased expression of epithelial marker E-cadherin (Fig. 5D and E).

**Figure 5:** Up-regulation of Shh in A549-M cells contributes to increased tumor cells migration and metastatic characteristics: A549-M cells were treated with Shh inhibitors such as Cyclopamine (2 µM) and GDC-0449 (20 nM) and assayed for wound healing (A), invasion (B) and clonogenic growth (C), and performed quantitative analysis showing attenuation of invasion by the treatment with Shh inhibitors. Western blot of A549-M cells before and after treatment with GDC-0449 (20 nM) for the expression of fibronectin (D). qRT-PCR for the expression of E-cadherin and ZEB1 mRNA in A549-M cells after treatment with GDC-0449 (20 nM) showing reversal of EMT phenotype compared to untreated A549-M cells (E). (*  =  *p*<0.05).

In order to further confirm the role of the induced expression of Shh by TGF-β1 in A549-M cells and its mechanistic association with increased cell migration, invasion and tumorigenesis, we knock-down the expression of Shh protein in A549-M cells by Shh-specific siRNA, and further assessed the transfection efficiency, which showed robust transfection efficiency (Fig. 6A). The knock-down of Shh protein in A549-M cells showed significant reduction in cell migration, invasion, and tumorigenic characteristics (Fig. 6B–D). The data clearly suggests the reversal of EMT morphology by the knock-down of Shh protein in A549-M cells (Fig. 6B inset). These data further confirmed that the inhibition in cell migration, invasion, and tumorigenic potential of A549-M cells is mechanistically mediated through the inhibition of Shh-mediated autocrine signaling.

**Figure 6:** Reduction in A549-M cells motility, invasiveness, and tumorigenesis by specific knock-down of Shh using Shh-specific siRNA: A549-M cells were transfected with Shh-specific siRNA (A): Transfection efficiency as assessed by GFP. The effect of knock-down of Shh was assessed by cell motility (wound healing) (B), invasion (C) and clonogenic growth (D) and further quantitated as detailed under “Materials and Methods” section, showing significant inhibition by Shh specific siRNA. (*  =  *p*<0.05).

### Down-regulation of Shh autocrine signaling in additional NSCLC cell lines led to the reduction in tumor cell migration, invasion, and tumorigenic characteristics

In order to further investigate whether the inhibition of Shh autocrine signaling leads to the reduction in cell migration, invasion, and tumorigenesis in other NSCLC cell lines that expresses Shh, we chose H1299 and H1650 cell lines, both of which were derived from lung metastasis of NSCLC patients. Both cell lines have been shown to be resistant to chemotherapy and targeted therapy (e.g. Erlotinib) [17], [38], [39]. Our results confirmed that both the cell lines expressed Shh as documented by qRT-PCR and Western blot analysis (Fig. 7A). Treatment of H1650 cells with Shh inhibitors GDC-0449 showed decreased cell migration, invasion and tumorigenic characteristics (Fig. 7B–C and Fig. S1), which clearly provide strong experimental support in favor of the role Shh in EMT phenotype. It is important to note that the treatment of H1650 cells with GDC-0449 led to the partial reversal of the EMT phenotype as documented by the reduced expression of fibronectin and ZEB1, and the increased expression of E-cadherin (Fig. 7D and E), which is consistent with the data in A549-M cells as presented under Fig. 5D and E. Moreover, these results are also consistent with the knock-down of Shh by Shh-specific siRNA in H1650 cells with robust transfection efficiency (Fig. 8A), and resulting in a significant reduction in cell migration and invasion (Fig. 8B and Fig. 8C). In addition, the treatment of H1299 cells with GDC-0449 or cyclopamine led to a significant reduction in invasion and tumorigenic behavior as assessed by clonogenic growth (Fig. S2A-B and Fig. S1). The treatment of H1299 cells with GDC-0449 also led to the partial reversal of the EMT phenotype as documented by reduced expression of fibronectin and ZEB1, and the increased expression of E-cadherin (Fig. S2C-D).

**Figure 7:** Down-regulation of Shh autocrine signaling in NSCLC cell lines led to the reduction in tumor cell migration, invasion, and tumorigenesis: A; both H1650 and H1299 cells expresses high levels of Shh mRNA compared to NHBE cells, and both cell lines have high Shh protein expression. B and C shows reduction in cell-invasion and the colony-forming ability of H1650 cells following treatment with Shh inhibitors such as GDC-0449 (20 nM). (D) Western blot of H1650 cells before and after treatment with GDC-0449 (20 nM) for the expression of fibronectin. (E) qRT-PCR for the expression of E-cadherin and ZEB1 mRNA in H1650 cells after treatment with GDC-0449 (20 nM) showing reversal of EMT compared to untreated H1650 cells. (*  =  *p*<0.05).

**Figure 8:** Down-regulation of Shh signaling in NSCLC cells lines (H1650 cells) leads to reduced cell motility and invasion. (A): Transfection efficiency was assessed by GFP. (B) Matrigel-Coated membrane assay where cells were labeled with DiIC1_2_ fluorescent dye. (C) Matrigel-Coated membrane assay where cells were labeled with immune-staining kit (Quik staining kit). (B and C right panel) also show quantitative data analysis. (*  =  *p*<0.05).

## Discussion

Previous studies have shown that the treatment of NSCLC cells (A549 cells) with TGF-β1 could induce EMT phenotype [13], [14], [16], a process that was originally reported to be involved in embryogenesis and gastrulation [4], [9], [40]. The induction of EMT in cancer cells confers these cells with the ability to become more motile and invasive with increased tumorigenic potential [4], [9], [11], [17], [18], [32], [33], [41]. Furthermore, the EMT phenotype appears to be involved in resistance to therapeutic agents. Thus, reversal of EMT by novel approaches may provide a tool by which one could enhance the effects of conventional therapeutic agents.

In this study, NSCLC cell lines (A549 and H2030) underwent EMT phenotypic changes (A549-M and H2030-M cells) after chronic exposure to TGF-β1, which was consistent with decreased expression of epithelial marker concomitant with increased expression of mesenchymal markers (Fig. 1A–C; Fig. 4A). In order to further characterize these cells, we assessed the ability of A549-M cells compared to A549 parental cells for cell migration, invasion and tumorigenic potential. Our data showed increased ability of A549-M cells for cell migration, invasion and tumorigenic potential compared to parental A549 cells (Fig. 2A–C). Interestingly, we also found that A549-M and H2030 cells showed high expression of Shh both at the mRNA and protein levels compared to parental cells (undetectable levels of Shh expression) (Fig. 3A–B; Fig. 4A). The up-regulation of Shh expression in A549-M cells is the first of its kind, which was also consistent with increased expression of GLI1 transcription factor, a downstream target gene of Hh signaling pathway (Fig. 3C–D) although the basal level of GLI1 expression was found to be high in the parental A549 cells. These results suggest that Hh signaling could be very active through non-canonical pathway (ligand-independence) in these cells. Our novel finding is very interesting not only because it connects two very important molecules of the developmental pathway such as TGF-β1 and Shh [42], [43] to tumor aggressiveness, but it is also consistent with published reports showing the role of EMT in tumor aggressiveness and metastasis [22], [25], [26], [31], [44]–[46]. However, no studies have shown the direct up-regulation of Hh ligand Shh mRNA and protein by TGF-β1 as documented in our current report although Shh has been reported to activate TGF-β family signaling through the ALK5-Smad 3 pathway in gastric cancer cells [21]. Moreover, it has been reported that TGF-β1 can induce GLI2 activation through Smad3 in pancreatic adenocarcinoma cell lines [47], and these published results suggest that there may exist a feed-back loop connecting TGF-β1 with Shh activation. Our finding also suggest that Hh signaling pathway reactivation in cancer epithelial cells within the tumor microenvironment could lead to the acquisition of aggressive phenotype of cancer cells within a tumor.

Although the mechanisms by which TGF-β1 can induce Hh ligand expression needs further investigation, our data clearly suggest that the activation of Shh signaling by TGF-β1 leads to increased tumor cell migration, invasion and tumorigenic potential of A549-M cells as documented by our mechanistic experiments using knock-down approach and by using chemical inhibitors of Shh signaling (Fig. 5A-C). Our results also suggest that the maintenance of EMT phenotype in A549-M cells may be related to the sustained activation of Hh. These results are also consistent with two other NSCLC cell lines that were derived from patients metastasis (H1650, H1299), and these two cell lines showed high basal levels of Shh expression, suggesting that lung metastatic cells have the ability to undergo EMT consistent with higher expression of Shh *in vivo*. Interestingly, the inhibition of TGF-β1-induced Shh signaling by pharmacological inhibitors or by siRNA decreased the ability of A549-M cells to migrate, invade and forming colony, and these results are consistent with previous reports showing that the activation of Shh signaling could increase invasion and metastasis [21], [23]–[26], [37], [44], [48].

We have also shown that the conditioned medium from A549-M cells has the ability to activate Shh downstream signaling in NIH 3T3 cells, which suggests that TGF-β1-induced EMT is mediated by the activation of Shh through both autocrine, paracrine or juxtacrine mechanisms although further mechanistic studies are warranted. Our results further showed the importance of Shh in EMT phenomenon, wherein inhibition of Shh signaling by GDC-0449 was able to down-regulate mesenchymal markers such as ZEB1 and fibronectin, which was consistent with up-regulation of epithelial marker such as E-cadherin (Fig. 5D and E and Fig. 7D and E). These results suggest that the attenuation of Shh signaling could reverse the EMT phenotype to mesenchymal-to-epithelial transition (MET) as shown in Fig. 6B (inset) where cells look more annular after Shh siRNA transfection, resulting in decreased cell migration, invasion and tumorigenic potential, which is consistent with the suggestion made by Feldmann et. al. [26]. More importantly, our data show for the first time that TGF-β1 induced EMT is mediated through up-regulation of Shh because knock-down of Shh by Shh specific siRNA significantly attenuated EMT induction by TGF-β1 treatment (Fig. 4B, C and D).

Clinically, NSCLC tumor tissues show higher levels of GLI1 expression compared to NSCLC cell lines [44], suggesting that the EMT phenotype with activated Shh signaling may be context-dependent such as what can be found in the tumor microenvironment where the tumor cells are chronically exposed to many factors including TGF-β1. This contention is partly supported by our data using four different NSCLC cell lines with epithelial vs. mesenchymal phenotype, and also suggested by a recently published report showing that chronic exposure to TGF-β1 in the tumor microenvironment may lead to the acquisition of EMT phenotype, which further leads to increased cell motility and invasiveness, resulting in tumor metastasis [46].

Based on existing evidence in the literature and our current data, we propose a model where epithelial tumor cells could be chronically exposed to TGF-β1 excreted by either stromal cells, immune cells or the tumor cells within the tumor microenvironment, resulting in the up-regulation of Shh both at the mRNA and at the protein levels and consequently causes activation of Hh signaling and the acquisition of EMT phenotype, which is responsible for tumor cell aggressiveness and metastasis (Fig. 9). Therefore, the inhibition of Shh signaling could be a useful approach for reducing tumor aggressiveness in NSCLC, and as such, the reversal of EMT could also be useful for re-sensitization of drug-resistant NSCLC to conventional therapeutics, which would likely contribute to the improved survival of patients who rightfully deserve better treatment outcomes.

**Figure 9:** Schematic diagram showing activation of TGF-β receptor by TGF-β1which leads to the up-regulation of Shh expression. The secreted Shh protein then activates Hh signaling pathway by inhibition of Patched (smoothened suppressor), which will repress smoothened, resulting in the activation of GLI1 and its translocation to the nucleus. GLI1 as a Hh transcription factor then could activate Hh target genes, which leads to the acquisition of EMT phenotype, and contributing to increased invasion, metastasis and drug resistance.

## Materials and Methods

### Cell Lines

The human lung adenocarcinoma cell lines, A549, H2030, H1299, H1650, and mouse fibroblast NIH-3T3 cells were purchased from the American Type Culture Collection (Manassas, VA) and maintained according to the American Type Culture Collection's instructions. The normal lung epithelial cell line (NHBE cells) was purchased from Lonza. NHBE cells where maintained and cultured according to Lonza's instructions. All the cell lines have been tested and authenticated using the Karmanos Cancer Center, Wayne State University's core facility (Applied Genomics Technology Center at Wayne State University) on March 13, 2009, and these authenticated cells were frozen for subsequent use. The method used for testing was short tandem repeat profiling using the PowerPlex 16 System from Promega. A549 cells were treated with TGF-β1 (5 ng/ml) for 21 days before experiments were conducted. Cells were treated with GDC-0449 (20 nM) or Cyclopamine (2 µM) for 72 hours, before conducting assays.

### Reagents and antibodies

Anti-Shh N-terminal peptide antibody and recombinant human TGF-β1 protein was purchased from R&D Systems (Minneapolis, MN). Cyclopamine was purchased from Sigma (San Louis, MO) and diluted in dimethyl sulfoxide (control vehicle). GDC-0449 (20 nM) was obtained from Genentech. Rabbit anti-GLI1 was purchased from Abcam. Rabbit anti-fibronectin was obtained from Santa Cruz biotechnology (CA, USA). Antibodies to glyceraldehyde 3-phosphate dehydrogenase (GAPDH) were purchased from Affinity BioReagents (Golden, CO.). Mouse anti-β-actin was obtained from Sigma (St. Louis, MO). β-tubulin rabbit mAb was obtained from cell signaling (Danvers, MA).

### Cell proliferation assay

Cells were treated with TGF-β1 for 21 days, Hh inhibitor for three-72 hour treatments, or knock-down with siRNA specific for Shh (si-Shh) for 48 hours. Prior to treatment, cells were seeded at 5×10^3^ cells per 100 µl of culture medium per well in 96-well plates. The number of viable cells was assessed in triplicate wells using a 3-(4,5-dimethylthiazol-2-yl)-2,5-diphenyltetrazolium bromide (MTT) assay (Sigma) according to the manufacturer's instructions. All assays were done in triplicates, and each experiment was repeated, at least, three times independently. Data reported here is one representative experiment.

### Wound healing assay

Cells were treated with TGF-β1 for 21 days, Hh inhibitor for three-72 hour treatments, or knock-down with siRNA specific for Shh (si-Shh) for 48 hours. Prior to treatment, cells were seeded at 1×10^6^ cells per well in a 6-well plates. Upon >90% confluence, cells were scraped across the cell monolayer using a plastic 200 µl tip. Photomicrographs were taken with Phase contrast objective microscope 4× magnification, at zero time point and after 24 hours. The measured ratio of the remaining wound area relative to the initial wound area was Quantified and reported. Quantification of the wound area using the NIH Image-J program was performed, and the results are expressed as the percentage of wound area change. Experiment was repeated at least three times, independently. Data reported here is one representative experiment.

### Matrigel invasion assay

Cells were treated with TGF-β1 for 21 days, Hh inhibitor for three-72 hour treatments, or knock-down with siRNA specific for Shh (si-Shh) for 48 hours. Following seeding cells at 5×10^4^ cells/well, invading cells at the bottom of the membrane and media in the lower chamber were detected by pre-labeled with DiIC1_2_ (3) Fluorescent Dye or by post-staining using immune-staining Diff-Quick™ staining kit after removal of noninvasive cells. Cells were seeded in the upper chamber of a 24-insert with serum-free medium. Upper chambers coated with Matrigel (fluoro-block insert and MATRIGEL™ Invasion Chamber; BD Biosciences, USA). Lower chamber contained 10% FBS plus regular media. After 24 h of incubation, invading cells were examined by using a fluorescence microscope and photographed. The transfection efficiency was photographed at 10X, whereas invading cells was photographed at 4× magnification. TECAN Ultra imaging system was used to measure the fluorescence of invading cells. Immune-stained cells were also counted under phase contrast objective microscope (10× magnification). The experiment was repeated at least three times independently. Data reported here is one representative experiment.

### Small interfering RNA (siRNA) transfection

Small interfering RNA (siRNA) specific for Shh (SHH Stealth RNAi™ siRNA) was purchased from Invitrogen. As a non-specific control siRNA, scrambled siRNA duplex was used which was also purchased from Invitrogen. Transfection was done using Lipofectamine RNAiMAX Transfection Reagent (Invitrogen) following the manufacturer's instruction. Experiment was repeated at least, three times independently. Data reported here is one representative experiment.

### Western blot analysis

Whole-cell protein extraction was conducted using RIPA buffer [50 mM Tris, 150 mM NaCl, 1%TritonX-100, 0.1% sodiumdodecyl sulfate and 1% Nadeoxycholate (pH 7.4)] supplemented with protease inhibitors (1 mMphenylmethylsulfonyl fluoride, 10 µg/ml peptasin A, 10 µg/ml aprotinin and 5 µg/ml leupeptin). Protein concentrations were then measured using Bio-Rad protein assay kits (Bio-Rad, Hercules, CA). Next, the protein lysates were resolved by sodium dodecyl sulfate–polyacrylamide gel electrophoresis (SDS-PAGE), then transferred onto nitrocellulose membranes (HybondTM-P; Amersham Biosciences, Piscataway, NJ), blocked with phosphate-buffered saline (PBS) containing 0.2% Tween 20 and 5% non-fat dry milk, incubated with primary antibody and then with horseradish peroxidase-labeled secondary antibody and developed using chemiluminiscent detection system, and the signals were then detected using X-ray film. Experiment was repeated at least three times independently. Data reported here is one representative experiment.

### Clonogenic assay

Cells were treated with TGF-β1 for 21 days, Hh inhibitor for three-72 hour treatments, or knock-down with siRNA specific for Shh (si-Shh) for 48 hours. Prior to treatment, cells were plated at a density of 1×10^3^ cells in 100-mm Petri dishes. Then the cells were incubated for 10–14 days at 37°C in a 5% CO_2_/5% O_2_/90% N_2_ incubator. Next, colonies were stained with 2% crystal violet and quantified using NIH Image-J software. The experiment was repeated at least three times independently. Data reported here is one representative experiment.

### Quantitative Real-time PCR

Quantitative real-time RT-PCR analysis was conducted; 1 µg of total RNA from each sample was subjected to reverse transcription using the High-Capacity RNA-to-cDNA Kit (Applied Biosystems) according to the manufacturer's protocol. Real-time PCR reactions were then carried out in a total volume of 25 µL reaction mixture (2 µL cDNA, 12.5 µL of 2 µL SYBR Green PCR Master Mix from Applied Biosystems, 1.5 µL of each 5 µmol/L forward and reverse primers, and 7.5 µL distilled H_2_O) using a SmartCycler II (Cepheid). The PCR program was started by 10 min at 95°C before 40 thermal cycles, each at 15 s at 95°C and 1 min at 60°C. Data were analyzed according to the comparative Ct method. Data was normalized by glyceraldehyde-3-phosphate dehydrogenase (GAPDH) expression in each sample. GLI1 primers have been previously described [25]. Shh primers (Shh-forward: GTGGCCGAGAAGACCCTA, Shh-reverse: CAAAGCGTTCAACTTGTCCTTA. GAPDH, ZEB1, and E-cadherin primers were previously described [49]. Experiment was repeated at least, three times independently. Data reported here is one representative experiment.

### Statistical analysis

The two-tailed v2 test was performed to determine the significance of the difference among the covariates. P values less than 0.05 were considered statistically significant. The SPSS software program (version 13.0, SPSS, Chicago, IL) was used for such analyses.

## Supporting Information

Figure S1 Shh signaling inhibition decreases tumorigenic potential of NSCLC cells. (A) clonogenic growth assay of three parental NSCLC cell lines compared to A549-M cells before and after treatment with Hh inhibitor GDC-0449 (20 nM), and (B) represent quantitative data analysis of the data presented in panel-A. (*  =  *p*<0.05).
(TIFF)

Figure S2 Inactivation of Shh by cyclopamine and GDC-0449 (20 nM) led to the reduction in tumor cell invasion (A), and tumorigenic potential (B) of H1299 NSCLC cell line. Right panel shows quantitative analysis. (C) Western blot of H1299 cells before and after treatment with GDC-0449 (20 nM) for the expression of fibronectin. (D) qRT-PCR expression of E-cadherin and ZEB1 mRNA of H1299 cells after treatment with GDC-0449 (20 nM) showing reversal of EMT compared to untreated H1299 cells. (*  =  *p*<0.05).
(TIFF)
